The article "Berberine and cinnamaldehyde together prevent lung carcinogenesis" was retracted in 2024. Reason: duplicated images.

# Berberine and cinnamaldehyde together prevent lung carcinogenesis

**DOI:** 10.18632/oncotarget.20059

**Published:** 2017-08-07

**Authors:** Mingjing Meng, Shengnan Geng, Zhenhua Du, Jingjing Yao, Yaqiu Zheng, Zibo Li, Zhenzhen Zhang, Jiahuan Li, Yongjian Duan, Gangjun Du

**Affiliations:** ^1^ Institute of Pharmacy, Pharmacy College of Henan University, Jinming District, Kaifeng, Henan Province 475004, China; ^2^ Department of Oncology, The First Hospital Affiliated to Henan University, Kaifeng, Henan Province 475001, China

**Keywords:** berberine, cinnamaldehyde, lung cancer, AMPK, AQP-1

## Abstract

Starving tumor cells by restricting nutrient sources is a promising strategy for combating cancer. Because both berberine and cinnamaldehyde can activate AMP-activated protein kinase (AMPK, a sensor of cellular energy status), we investigated whether the combination of berberine and cinnamaldehyde could synergistically prevent lung carcinogenesis through tumor cell starvation. Urethane treatment induced lung carcinogenesis in mice, downregulated AMPK and mammalian target of rapamycin (mTOR) while upregulating aquaporin-1 (AQP-1) and nuclear factor kappa B (NF-κB). Together, berberine and cinnamaldehyde reduced mouse susceptibility to urethane-induced lung carcinogenesis, and reversed the urethane-induced AMPK, mTOR, AQP-1, and NF-κB expression patterns. *In vitro*, berberine and cinnamaldehyde together induced A549 cell apoptosis, prevented cell proliferation, autophagy, and wound healing, upregulated AMPK, and downregulated AQP-1. The effects of the combined treatment were reduced by rapamycin (a mTOR inhibitor) or HgCL_2_ (an AQP inhibitor), but not Z-VAD-FMK (a caspase inhibitor). The berberine/cinnamaldehyde combination also prevented A549 cell substance permeability and decreased intracellular ATP concentrations. These results suggest the combination of berberine and cinnamaldehyde limited both primary and adaptive nutrient acquisition by lung tumors via AMPK-reduced AQP-1 expression, which ultimately starved the tumor cells.

## INTRODUCTION

Despite improvements in screening and patient care, cancer remains a leading cause of death worldwide [1]. Systemic therapies, such as chemotherapy and hormone therapy, are standards of care in the management of many cancer types. However, systemic therapeutic-associated toxicity is common, and novel, low-toxicity anti-cancer therapeutic drugs are needed [2]. Natural products, including herbs and spices, have been used for millennia to prevent or treat various human diseases, including cancer [3]. Plants are an abundant source of phytochemicals that show potential as anti-cancer therapeutics [4]. However, the cancer preventive effects of single agents are frequently limited. Jiao Tai Wan (JTW), which contains *Rhizoma coptidis* (the whole plant) and *Cortex cinnamomi* (bark of the plant), is a common remedy for insomnia that was developed during the Ming Dynasty [5] and was recently used to treat clinical diabetes [5]. *R. coptidis* and its major constituent, berberine, and *C. cinnamomi* and its major constituent, cinnamaldehyde, exhibit anti-cancer activities [6–7]. Therefore, JTW or a combination of berberine and cinnamaldehyde may be efficacious in preventing cancer.

The article "Berberine and cinnamaldehyde together prevent lung carcinogenesis" was retracted in 2024. Reason: duplicated images.

Tumor cell starvation via nutrient restriction is a promising strategy to combat cancer [8]. An alternative strategy to achieve both therapeutic selectivity and efficiency is to take advantage of fundamental biochemical and metabolic differences between cancer cells and normal cells [9]. Increased metabolic rates and suppressed osmotic functions may lead to nutrient deficiency in tumor cells. We previously showed that tumor interstitial fluid provides better nutrition for the tumor than angiogenesis [8]. The AMP-activated protein kinase (AMPK), an important downstream effector of the tumor suppressor liver kinase 1 (LKB1), senses cellular energy status and inhibits tumorigenesis [10, 11]. However, its role in cancer progression has not been well characterized. Because both berberine and cinnamaldehyde can activate AMPK [11, 12], we hypothesized that these compounds together may reduce cancer cell nutrient intake and ultimately starve the cells. Thus, the present study investigated the cancer preventive effects of the combination of berberine and cinnamaldehyde and explored the molecular mechanisms underlying these effects.

## RESULTS

### Berberine and cinnamaldehyde together prevent urethane-induced lung carcinogenesis

Combinations of various phytochemicals derived from dietary sources or medicinal plants not only may reduce the risks of specific cancers, but also have been shown to suppress cancer cell proliferation [13]. Urethane-induced epithelial carcinogenesis results in histological and molecular changes that resemble human lung cancer and allows for mechanistic evaluations of therapeutic interventions during tumor development [14]. In mice with urethane-induced lung carcinoma, oral administration of berberine and cinnamaldehyde in combination induced lean body phenotypes in the combination group (32.7 ± 2.8 g, *P* < 0.05) compared to the UC group (36.8 ± 2.6 g), which was not significantly different from the normal (37.3 ± 2.5 g; *P* > 0.05), berberine (35.9 ± 2.7 g; *P* > 0.05), cinnamaldehyde (33.5 ± 2.6 g; *P* > 0.05), and JTW (34.2 ± 2.8 g; *P* > 0.05) groups (Figure 1A).

The article "Berberine and cinnamaldehyde together prevent lung carcinogenesis" was retracted in 2024. Reason: duplicated images.

**Figure 1:** Berberine and cinnamaldehyde together prevented urethane-induced lung carcinogenesis Body weight at the beginning (d 1) and end (26 weeks) of the experiment (**A**). Lung carcinoma incidence and number (**B**) and multiplicity (average neoplastic nodules per lung) (**C**). The normal group included non-carcinogenic mice fed in parallel, and the UC group included untreated carcinogenic mice. *P < 0.05, **P < 0.01 *vs* UC.

To determine whether the compounds and herbs resulted in toxicity, we examined cumulative food intake, autonomic activity, liver and renal function, and hematological parameters during the final week. Consistent with reduced body weights, the cinnamaldehyde and the combination-treated mice consumed less food than the UC group (29.3 ± 5.0, 26.7 ± 4.4, 24.2 ± 4.9, and 33.1 ± 4.2 g/mouse weekly in the berberine, cinnamaldehyde, combination, and UC groups, respectively). However, no differences were observed in autonomic activity and levels of liver transaminases, creatinine, and hematological factors between the UC and treatment groups (data not shown), indicating no berberine or cinnamaldehyde toxicity in mice.

In contrast to the UC group, berberine or cinnamaldehyde treatment alone only prevented lung carcinoma incidence (75%, 90%, and 100% in the berberine, cinnamaldehyde, and UC groups, respectively) and multiplicity (15.3 ± 2.4 (*P* < 0.01) and 18.2 ± 2.5 (*P* < 0.01) in the berberine and cinnamaldehyde groups, respectively, vs. 21.4 ± 3.5 in the UC group) to some extent, whereas the combination of berberine and cinnamaldehyde or JTW reduced lung carcinogenesis susceptibility (carcinoma incidences of 35%, 30%, and 100% in the JTW, combination, and UC groups, respectively, and multiplicities of 8.3 ± 2.6 (*P* < 0.001) and 7.5 ± 2.2 (*P* < 0.001) in the JTW and combination groups, respectively, vs. 21.4 ± 3.5 in the UC group) (Figure 1B–1C) regardless of tumor histological heterogeneity.

### Berberine and cinnamaldehyde together regulate inflammation and oxidative stress during carcinogenesis

We analyzed correlations between the serum inflammation markers, IL-1, IL-6, high-sensitivity C-reactive protein (hs-CRP), and tumor necrosis factor α (TNF-α), and oncogenesis and between the serum oxidative stress marker, 8-hydroxy-2’-deoxyguanosine (8-OHdG), and oncogenesis at 26 weeks. Serum IL-1, IL-6, hs-CRP, and TNF-α levels were decreased in the berberine (*P* < 0.01) and cinnamaldehyde (*P* < 0.01) groups compared to the UC group, which had higher serum inflammation marker levels than the normal group, indicating a positive correlation between inflammation and lung cell oncogenesis (Figure 2A–2D). Compared to the UC group, serum interferon gamma (IFN-γ) and interleukin-2 (IL-2) (the type 1 immunostimulatory cytokines) levels were decreased in the berberine group (*P* > 0.05), but increased in the cinnamaldehyde group (*P* < 0.01), whereas serum IL-4 and IL-10 (type 2 immunoinhibitory cytokines) levels were increased in the berberine group (*P* < 0.01), but decreased in the cinnamaldehyde group (*P* < 0.01) (Figure 3A–3D), indicating an immune regulatory difference between berberine and cinnamaldehyde. However, JTW or the combination of berberine and cinnamaldehyde had serum IL-4, IL-10, IFN-γ, and IL-2 levels similar to those of the normal group (Figure 3), indicating a therapeutic advantage of the herbs and combined compounds. Consistently, serum 8-OHdG and reactive oxygen species (ROS) levels were only decreased to a small extent in the berberine and cinnamaldehyde groups compared to the UCgroup, which had higher levels than the normal group, indicating a positive correlation between oxidative stress and lung cell oncogenesis. However, serum 8-OHdG and ROS levels were suppressed in the combination and JTW groups (Figure 4A–4B). Additionally, JTW or the combination of berberine and cinnamaldehyde enhanced lung epithelium integrity as indicated by evans blue permeability and lung water content, which was only slightly reduced by berberine or cinnamaldehyde alone (Figure 4C–4D).

The article "Berberine and cinnamaldehyde together prevent lung carcinogenesis" was retracted in 2024. Reason: duplicated images.

**Figure 2:** Berberine and cinnamaldehyde together decreased inflammation during carcinogenesis Berberine and cinnamaldehyde together or JTW decreased inflammation as indicated by increased serum IL-1 (**A**), IL-6 (**B**), hs-CRP (**C**), and TNF-α (**D**) levels (*n* = 5). *P < 0.05, **P < 0.01 *vs* UC.

**Figure 3:** Berberine and cinnamaldehyde together regulated immunity during carcinogenesis Berberine and cinnamaldehyde together or JTW regulated immunity as indicated by serum levels of the type 1 immunostimulatory cytokines, IFN-γ (**A**) and IL-2 (**B**), and type 2 immunoinhibitory cytokines, IL-4 (**C**) and IL-10 (**D**) (*n* = 5). *P < 0.05, **P < 0.01 *vs* UC.

**Figure 4:** Berberine and cinnamaldehyde together decreased oxidative stress and lung epithelium integrity Berberine and cinnamaldehyde together decreased oxidative stress as indicated by increased serum 8-OHdG (**A**) and ROS (**B**) levels, and lung epithelium integrity as indicated by evans blue permeability (**C**) and lung water content (**D**) (*n* = 5). *P < 0.05, **P < 0.01 *vs* UC.

### Berberine and cinnamaldehyde together regulate lung signaling protein levels during carcinogenesis

To explore why berberine and cinnamaldehyde together reduced lung carcinogenesis susceptibility, we examined urethane-associated changes in cellular signaling via western blot analyses at 26 weeks. AMPK and mTOR in the lung were only slightly upregulated in the berberine and cinnamaldehyde groups (*P* < 0.05) compared to the UC group, which exhibited lower AMPK and mTOR levels than the normal group (*P* < 0.01), indicating autophagy as the primary nutrient acquisition method in these two treatment groups (Figure 5A). JTW or the combination of berberine and cinnamaldehyde upregulated AMPK and mTOR (*P* < 0.001). On the contrary, NF-κB and aquaporin-1 (AQP-1) in the lung were only slightly downregulated in the berberine and cinnamaldehyde groups (*P* < 0.05) compared to the UC group, which exhibited higher NF-κB and AQP-1 levels than the normal group (*P* < 0.01), indicating influx of exogenous nutrients as the primary nutrient acquisition method in these two treatment groups. JTW or the combination of berberine and cinnamaldehyde downregulated NF-κB and AQP-1 (*P* < 0.001).

The article "Berberine and cinnamaldehyde together prevent lung carcinogenesis" was retracted in 2024. Reason: duplicated images.

**Figure 5:** Berberine and cinnamaldehyde together regulated lung signaling protein expression during carcinogenesis Berberine and cinnamaldehyde together regulated AMPK, mTOR, NF-κB, and AQP-1 expression as indicated by western blotting (**A**), and promoted lung epithelial cell proliferation as indicated PCNA, EMT, and N-cadherin upregulation and E-cadherin downregulation as shown by IHC (**B** and **C**). Assays were performed in triplicate. *P < 0.05, **P < 0.01 *vs* UC.

### Berberine and cinnamaldehyde together prevent lung epithelial cell proliferation and EMT during carcinogenesis

Carcinogenesis is the final result of epithelial proliferation and the epithelial to mesenchymal transition (EMT) [15, 16]. To verify the effects of the herbs and combined compounds on cancer prevention, we also examined urethane-associated changes in lung epithelial cell proliferation and EMT via immunohistochemistry (IHC) at 26 weeks. Proliferating cell nuclear antigen (PCNA), a lung epidermal cell proliferation marker, was only slightly downregulated in the berberine and cinnamaldehyde groups, but was suppressed in the JTW and combination groups compared to the UC group, which exhibited higher levels than the normal group (Figure 5B–5C). Similarly, lung EMT, as indicated by E-cadherin and N-cadherin levels, was also only slightly decreased in the berberine and cinnamaldehyde groups, but was suppressed in the combination and JTW groups compared to the UC group, which exhibited higher levels than the normal group (Figure 5B–5C).

### Berberine and cinnamaldehyde together lead to A549 cell starvation

We treated A549 cells *in vitro* with berberine and cinnamaldehyde alone or in combination to observe cell proliferation, autophagy, and wound healing. MTT assay results showed that berberine or cinnamaldehyde alone only slightly reduced cell proliferation, while their combination suppressed cell proliferation in a time-dependent manner (Figure 6A). Similarly, berberine and cinnamaldehyde together increased cell apoptosis more than either compound alone (Figure 6B–6C). However, berberine or cinnamaldehyde alone stimulated cell autophagy as indicated by autophagosome and LC3-B production under 10% serum culture conditions, indicating a cell starvation state. Autophagy under these conditions could be aborted by treatment with berberine and cinnamaldehyde together (Figure 7A). Compared to untreated cells, 2% serum-induced cell autophagy (Figure 7B) and wound healing (Figure 8) were decreased in the berberine group (*P* > 0.05), but were not affected in the cinnamaldehyde group (*P* < 0.01), whereas berberine and cinnamaldehyde together suppressed both.

The article "Berberine and cinnamaldehyde together prevent lung carcinogenesis" was retracted in 2024. Reason: duplicated images.

**Figure 6:** Berberine and cinnamaldehyde together suppressed A549 cell proliferation and promoted apoptosis (*n* = 3) (B) and (C) in a time-dependent manner *(n* = 6) (A) *P < 0.05, **P < 0.01 *vs* control

**Figure 7:** Berberine and cinnamaldehyde together suppressed A549 cell autophagy Berberine and cinnamaldehyde together aborted berberine- or cinnamaldehyde-induced cell autophagy under 10% serum culture conditions (*n* = 3) (**A**). Combination therapy suppressed autophagy under 2% serum culture condition (*n* = 3) (**B**). Cells in the AO staining group were in the early stage of culture medium replacement. Cells in the LC3-B staining group were harvested at a late cell culture stage. *P < 0.05, **P < 0.01 *vs* control.

**Figure 8:** Berberine and cinnamaldehyde together suppressed wound healing in A549 cells *P < 0.05, **P < 0.01 *vs* control.

We also found that the effects of berberine and cinnamaldehyde together were suppressed by pre-treatment with the mTOR inhibitor, rapamycin, or the aquaporin inhibitor, HgCl_2_, but were unaffected by the caspase inhibitor, Z-VAD-FMK (Figures 6 and 8). The combination of berberine and cinnamaldehyde synergistically increased AMPK and decreased AQP-1 levels (Figure 9A). Additionally, the two compounds together reduced cell substance permeability (Figure 9B) and intracellular ATP concentrations (Figure 9C), indicating cancer cell starvation.

**Figure 9:** Berberine and cinnamaldehyde together synergistically regulated AMPK/AQP-1 protein levels and prevented substance permeability in A549 cells Berberine and cinnamaldehyde together upregulated AMPK and downregulated AQP-1 (*n* = 3) (**A**), prevented substance permeability as indicated by increased intracellular rhodamine B (*n* = 3) (**B**), and decreased intracellular ATP concentrations (*n* = 3) (**C**) *P < 0.05, **P < 0.01 *vs* control.

The article "Berberine and cinnamaldehyde together prevent lung carcinogenesis" was retracted in 2024. Reason: duplicated images.

## DISCUSSION

Approaches to reducing the global cancer burden include two major strategies: active prevention and early therapeutic intervention [17]. Herb combinations have been used to treat human illnesses as part of Chinese phytotherapy for millennia [18]. Recent studies indicate that traditional Chinese medicine (TCM)-based treatments might prevent tumorigenesis, shrink or stabilize tumors, and reduce tumor recurrence and metastasis [19]. In this study, we assessed the cancer preventive effects of berberine and cinnamaldehyde together or JTW. Our results suggest that the combination of berberine and cinnamaldehyde prevents lung carcinogenesis via AMPK-reduced AQP-1 expression, which ultimately starves tumor cells. Ours is the first report describing the efficacy and molecular mechanisms of berberine and cinnamaldehyde together in preventing lung cancer.

Development of cancer preventive agents is often similar to development of therapies to treat advanced cancers [20], and both strategies may focus on mediating cancer-predisposing conditions [21]. Cancer cells use higher nutrient amounts than non-cancer cells to support the bioenergetic and biosynthetic demands of increased proliferation. While cancer cell constitutive anabolism supports proliferation, tumor cells also become reliant on a steady influx of exogenous nutrients [23]. Thus, reducing access to nutrients may effectively and selectively limit tumor cell growth. Previously, starvation strategies and agents aimed to limit specific substrates based on metabolic differences between normal and transformed cells [22]. However, tumor heterogeneity can limit starvation agent efficacies, because primary nutrient limitation may stimulate adaptive nutrient acquisition [23]. Therefore, ideal tumor starvation strategies limit both primary and adaptive nutrient acquisition [24].

AMPK is involved in various energy-intensive pathological processes, such as inflammation and apoptosis [25]. AMPK is an evolutionarily conserved energy sensor with central roles in maintaining energy homeostasis [25–27], and is a downstream activator of the tumor suppressor, liver kinase B1 (LKB1). AMPK activation reportedly suppresses cell proliferation in many tumor types by regulating cell cycle progression or inhibiting protein synthesis [28]. Aquaporins are permeable to water and low-molecular weight solutes, such as glycerol and urea [29], and AQP-1 is important for liquid exchange between alveoli and capillaries [30]. AQP-1 is a prognostic factor for many cancer types [31], and AMPK activation suppresses AQP-9 [32]. However, whether AMPK and AQP-1 have roles in lung carcinogenesis and whether AMPK also suppresses AQP-1 remained unclear.

The article "Berberine and cinnamaldehyde together prevent lung carcinogenesis" was retracted in 2024. Reason: duplicated images.

This study compared the efficacies of berberine and cinnamaldehyde alone and in combination as cancer preventives. We treated mice with 100 mg/kg body weight berberine or 5 mg kg body weight cinnamaldehyde, or a combined dose of 105 mg/kg body weight at a ratio of 20:1 berberine:cinnamaldehyde. We found that the combination treatment or JTW prevented urethane-induced lung carcinogenesis and regulated inflammation and oxidative stress during carcinogenesis. We noted lung congestion in the berberine and combination treatment groups, but not other groups, and this may have been associated with berberine-stimulated heat dissipation during urethane-induced lung carcinogenesis. We also found that JTW or the combination treatment upregulated AMPK and mTOR, but downregulated NF-κB and AQP-1 in the lung during carcinogenesis, suggesting that treatment restored urethane-disrupted signal transduction pathways. Finally, we showed that JTW or the combination treatment prevented lung epithelial cell proliferation and EMT during carcinogenesis. The accumulated publication had shown that the function of AMPKalpha1, AMPKalpha2 and LKB1 in carcinogenesis was controversial [33, 34, 35]. Our results suggest that AMPK, regardless of subtype, and AQP-1 play opposite roles in lung carcinogenesis and that lung cancer prevention via berberine and cinnamaldehyde is associated with these two proteins. Inconsistent with previous reports, urethane downregulation of AMPK did not activate mTOR, but instead suppressed it. JTW or the combination of berberine and cinnamaldehyde upregulated AMPK and mTOR, indicating that autophagy and exogenous nutrient influx acted synergistically during carconogenesis.

In traditional JTW, the amount of *R. coptidis* is greater than that of *C. cinnamomi*, and recent findings suggest that this ratio has important implications for clinical practice [36]. The ratio of *R. coptidis* (whole plant) to *C. cinnamomi* (bark only) traditionally used to treat insomnia was 10:1 (w/w) [37], but a 2:1 (w/w) ratio has been commonly applied to treat diabetes in recent practice [38]. The optimal *R. coptidis* to *C. cinnamomi* ratio for cancer prevention is unknown. Before beginning the present study, we established three JTW formulations with *R. coptidis: C. cinnamomi* ratios of 2:1, 1:1, and 1:2 (w/w), and compared the cancer preventive efficacies of these formulations in a urethane-induced lung carcinoma model. Mice lost weight and showed no satiety in the 1:1 ( < 15% normal body weight) and 2:1 ( > 15% normal body weight) groups, and satiety and weight loss ( > 20% normal body weight) in the 1:2 group (data not shown). Therefore, we selected 1:1, *R. coptidis*: *C. cinnamomi* and 20:1, berberine: cinnamaldehyde formulations for use in the present study. The combination therapies prevented A549 cell proliferation, autophagy, and wound healing via AMPK upregulation and AQP-1 downregulation. However, these effects were suppressed by the mTOR inhibitor, rapamycin, or the aquaporin inhibitor, HgCl_2_, but not the caspase inhibitor, Z-VAD-FMK. The combination therapies also decreased substance permeability and intracellular ATP levels, and promoted cell apoptosis. These results together indicate starvation-related cell death.

The article "Berberine and cinnamaldehyde together prevent lung carcinogenesis" was retracted in 2024. Reason: duplicated images.

Our *in vitro* conclusions are limited by the fact that we tested the therapies in only one cell line. However, we compared AMPK and AQP-1 expression in A549 and L929 cells (an embryonic lung fibroblast cell line), and observed lower AMPK and higher AQP-1 levels in A549 cells compared to L929 cells (data not shown). These findings support our hypothesized negative feedback relationship between the two proteins.

Certain types of cancer may be defined as chronic diseases, similar to hypertension and diabetes [39, 40]. Recent findings indicate that TCM application could provide benefit over the entire cancer treatment course [18]. However, the complexity of TCM components limits their application. Although limiting nutrient access is a feasible alternative approach to blocking anabolism in cancer cells, tumor heterogeneity is an obstacle to good outcomes, including for those therapies targeting specific metabolic pathways [23]. However, the novel combination of berberine and cinnamaldehyde limits both primary and adaptive nutrient acquisition in tumors, thus potentially preventing tumor adaptation. Thus, JTW and the combination of berberine and cinnamaldehyde are potentially efficacious strategies for tumor cell starvation.

## MATERIALS AND METHODS

### Materials

JTW was purchased from the First Affiliated Hospital of the Henan University of Chinese Medicine. Each JTW packet contained 1 g of concentrated *R. coptidis* granules (equal to 3 g *R. coptidis*) and 1 g of *C. cinnamomi* concentrated granules (equal to 3 g *C. cinnamomi*). *R. coptidis* concentrated granules contain high amounts of berberine (100.0 mg/g via high-performance liquid chromatography (HPLC)). *C. cinnamomi* concentrated granules were mainly composed of cinnamaldehyde (5.0 mg/g via HPLC). Cinnamaldehyde (purity > 98% via HPLC) and berberine (purity > 98% via HPLC) were purchased from Yiji Industrial Co., Ltd. (Shanghai, China). Urethane, Z-VAD-FMK, rapamycin, HgCL_2_, AO and evans blue were purchased from Sigma Chemical Co (St.Louis. MO. USA). Antibodies used included anti-PCNA, anti-AMPK, anti-mTOR, anti-NF-κB, anti-AQP1, anti-E-cadherin, anti-N-cadherin, anti-LC3-B, anti-glyceraldehyde-phosphate dehydrogenase (GAPDH), and anti-β-actin were obtained from BD Pharmingen. Horseradish peroxidase (HRP)-conjugated goat anti-mouse IgG polyclonal antibody, peroxidase substrate DAB (3, 3′-diaminobenzidine) were obtained from Nichirei Bioscience (Tokyo, Japan). Annexin V-FITC / PI Apoptosis Detection Kit was obtained from Solarbio (Beijing, China). 5-HIAA ELISA assay kit, Mouse quantitative ELISA kits (IFN-γ, IL-2, IL-1, IL-4, IL-6, IL-10, TNF-α, hs-CRP, ROS, and 8-OHdG) were obtained from R&D Systems. Standard rodent chow was purchased from Henan Provincial Medical Laboratory Animal Center (Zhengzhou, China), License No. SCXK (YU) 2015-0005, Certificate No. 41000100002406.

The article "Berberine and cinnamaldehyde together prevent lung carcinogenesis" was retracted in 2024. Reason: duplicated images.

### Animals

Cohorts of 5- to 6-week-old female ICR mice were obtained from Henan Provincial Medical Laboratory Animal Center. All mice were housed in individual ventilated cages under a 12-h light-dark cycle (lights on 7:00 AM to 7:00 PM). Animals were fed standard rodent chow and water. All animal procedures were approved by the Animal Experimentation Ethics Committee of Henan University (permission number HUSAM2014-216), and all procedures were performed in strict accordance with the Guide for the Care and Use of Laboratory Animals and the Regulation of Animal Protection Committee to minimize suffering and injury. Animals were monitored daily and were euthanized via carbon dioxide overdose at the end of the experiment or at the first sign of shortness of breath, reduced locomotion, or reduced body weight (> 30% total body weight). All surgeries were performed under general anesthesia induced via intraperitoneal injection of 45 mg/kg pentobarbital sodium, and all efforts were made to minimize suffering.

### Urethane-induced lung adenocarcinoma model

ICR mice were administered freshly prepared urethane to induce lung adenocarcinomas as previously described [41]. Mice received an intraperitoneal injection of urethane (600 mg/kg body weight) dissolved in sterile 0.9% NaCl once weekly for 10 weeks. Following urethane injection, mice were randomly divided into six groups (normal; urethane/control; urethane/berberine (100 mg/kg body weight); urethane/cinnamaldehyde (5 mg/kg body weight); urethane/combination (berberine: cinnamaldehyde = 20:1, 105 mg/kg body weight); urethane/JTW (2 g/kg body weight)). Dose selection was based on doses reported in a pilot experiment [42, 43, 44, 45]. Mice in the control and treated groups were intraperitoneally injected with urethane, and animals in the normal group were treated only with vehicle (normal saline). Following the first urethane injection, treated mice received therapeutic drugs alone or in combination via intragastric administration (all therapeutic drugs were suspended in 0.1% (v/v) aqueous Tween-80 for animal administration) once daily for 25 weeks. Food and water were provided ad libitum during the study. The health of the mice was monitored daily, and body weights were measured weekly. At 26 weeks after the first urethane injection, orbital venous blood was collected for plasma 5-HIAA assay using an ELISA kit. Mice were sacrificed under anesthesia with pentobarbital sodium (45mg/kg), lung carcinoma incidence and multiplicity (average carcinomas per mouse) were determined, and lungs were biochemically processed.

The article "Berberine and cinnamaldehyde together prevent lung carcinogenesis" was retracted in 2024. Reason: duplicated images.

Each study group included 25 mice. Mice not challenged with urethrane were “normal,” and challenged mice were “UC.” At the end of the experiment, there were 20 mice per group. Mice with clear evidence of myocardial infarction were excluded from the study and euthanzed. The endpoint of the experiment was the first sign of shortness of breath, reduced locomotion, or reduced body weight ( > 30% total body weight) because of lung tumors.

### Clinical chemistry

Blood samples were collected for chemical analyses from the orbital venous plexus at the time of sacrifice after 6 h of fasting. IFN-γ, IL-2, IL-1, IL-4, IL-10, IL-6, hs-CRP, and TNF-α serum concentrations were determined using a plate reader (Mulitiskan Go 1510, German) according to the manufacturer's protocol. Results were calculated from linear curves obtained using the Quantikine kit standards.

### Oxidative stress analysis

Serum 8-hydroxy-2’-deoxyguanosine (8-OHdG) levels were measured using an ELISA assay kit. Serum ROS levels, a marker of oxidative stress, were also determined using an ELISA assay kit according to the manufacturer's protocol. The complete assay procedure was similar to clinical chemistry methods.

### Immunohistochemistry

For IHC analyses, serial sections (5 μm) of lung were cut and attached to superfrost plus microscope slides. Slides were warmed at 60°C for 1 h, deparaffinized in xylene, and dehydrated in decreasing concentrations of ethanol. After blocking with 3% hydrogen peroxide for 10 min, sections were incubated with 0.1% TritonX-100 in PBS for 20 min at room temperature, and then immersed in a 5% bovine serum albumin (BSA) blocking solution for 20 min at room temperature. Sections were then incubated with primary antibodies (diluted to 1% with antibody diluent) against PCNA, E-cadherin, or N-cadherin overnight at 4°C. Antigen–antibody binding was detected using a rabbit IgG IHC kit. Signal was developed using the peroxidase substrate, DAB, which appears as a brown reaction product. All sections were counterstained with hematoxylin and were imaged under a microscope. Two pathologists interpreted the IHC results using a semi-quantitative histological score (HSCORE), as described previously [46].

The article "Berberine and cinnamaldehyde together prevent lung carcinogenesis" was retracted in 2024. Reason: duplicated images.

### Lung epithelium integrity and lung water content

The integrity of the lung epithelium was assayed using the EB dye extra-barrier technique as previously described [46]. Lung water content was measured as previously described [46].

### Western blot analysis

Lung or A549 cells extracts were prepared in radio immunoprecipitation assay (RIPA) cell lysis buffer. Equal amounts of protein were separated via 12% sodium dodecyl sulfate-polyacrylamide gel electrophoresis, electroblotted on nitrocellulose membranes, and probed with antibodies against AMPK, mTOR, NF-κB, AQP-1, β-actin or GAPDH. Antibody binding was detected via enhanced chemiluminescence according to the manufacturer's instructions (Pierce, Rockford, IL). Band density was quantified using ImageJ software (NIH, Bethesda, MD, USA) and normalized to the corresponding control group.

### Cell culture

The human alveolar basal epithelial cancer cell line, A549, was grown in RPMI 1640 medium supplemented with 10% (v/v) FBS. Cells were grown in a humidified atmosphere containing 5% CO_2_ and 95% air at 37°C. For *in vitro* experiments, 50 mM berberine and cinnamaldehyde stock solutions (in DMSO, stored at –20°C) were diluted in cell culture medium to working concentrations. The maximum final DMSO concentration was < 0.1% for each treatment. DMSO was used as a control.

### Cell proliferation

A549 cells (1 × 10^4^ cells/well) were incubated in a 96-well plate overnight at 37°C. Cells were treated with specified concentrations of berberine and cinnamaldehyde alone or in combination in the presence or absence of 50 μM Z-VAD-FMK, 20 μM rapamycin, or 100 μM HgCL_2_, which were tolerated by cells without morphological alterations or signs of death. Each condition was tested in six replicates. During the final 4 h of the 72-h incubation, supernatants were discarded and 100 μL MTT (0.5 mg/ml) was added to each well. After 4 h, MTT was discarded and 100 μL DMSO was added to each well. Absorbance at 570 nm was determined using a plate reader (Elx-800; Bio-Tek, USA). Cell proliferation assay results are presented as a percentage of the control cells.

### Cell apoptosis and autophagy detection

Cell apoptosis was evaluated using propidium iodide (PI)/Annexin V-FITC fluorescence staining. Briefly, A549 cells were treated with specified concentrations of berberine and cinnamaldehyde alone or in combination for 48 h in the presence or absence of Z-VAD-FMK, rapamycin, or HgCL_2_. 5 μl PI and 5 μl Annexin V-FITC were added to cells for 10 min, and then washed once with PBS. After staining, cells were visualized and analyzed using a Cellometer K2 (Nexcelom Bioscience).

The article "Berberine and cinnamaldehyde together prevent lung carcinogenesis" was retracted in 2024. Reason: duplicated images.

To assess cell autophagy, A549 cells were treated with specified concentrations of berberine and cinnamaldehyde alone or in combination for 48 h under 10% serum or 2% low serum culture conditions. Cells were stained with AO (1 μg/ml) at 37°C for 30 min before observation. Red acidic vesicular organelles (AVOs) stained by AO in autophagic cells were visualized under a fluorescence microscope. Cell autophagy was further estimated via LC3-B immunofluorescent staining using PE-conjugated anti-LC3-B. Intracellular fluorescence was estimated using flow cytometry assay.

### Wound-healing assay

A549 cells (3 × 10^4^ cells/well) were seeded into a 24-well plate and cultured to confluence. The monolayer was then scratched with a 200-μL pipette tip to create an approximately 1 mm-wide wound area, and was washed twice with PBS to remove floating cells. Cells were then treated with specified concentrations of berberine and cinnamaldehyde alone or in combination for 48 h in the presence or absence of Z-VAD-FMK, rapamycin, or HgCL_2_ under 2% serum culture conditions. Wounded monolayer images were obtained using a microscope. Wound repair rates were expressed as the gap percentage relative to the total area of the cell-free region immediately after the scratch was generated, according to image analysis software (Olympus, Tokyo, Japan).

### Substance permeability assay

Substance permeability was estimated by calculating the amount of rhodamine B dye that passed through the samples over different time intervals. Intracellular rhodamine B fluorescence was measured using flow cytometry.

### Intracellular ATP assay

Intracellular ATP was measured using the luciferin/luciferase system. Briefly, A549 cells were treated with specified concentrations of berberine and cinnamaldehyde alone or in combination for 48 h. Cell membranes were permeabilized using 100 μl somatic cell ATP releasing reagent (Sigma-Aldrich Co., St Louis, MO) and were then reacted with 100 μl ATP assay mix reagent containing 0.28 mg/ml luciferin and 1 mg/ml luciferase. After 10 min incubation at room temperature, luminescence was measured over a 0.5 s integration time using a luminometer. Intracellular ATP level was expressed as the percentage of the luminescence intensity of the control cells.

### Statistical analyses

A Shapiro-Wilk test was carried out to test for normal distributions. Normally distributed data are presented as means ± SD and were statistically analyzed using GraphPad Prism, Version 5.0 (San Diego, CA, USA). Differences among groups were evaluated using a one-way analysis of variance (ANOVA). *P* < 0.05 was considered statistically significant.

The article "Berberine and cinnamaldehyde together prevent lung carcinogenesis" was retracted in 2024. Reason: duplicated images.

## References

[1] Jemal A, Bray F, Center MM, Ferlay J, Ward E, Forman D (2011). Global cancer statistics. CA Cancer J Clin.

[2] Horwich A (2006). Systemic treatment for prostate cancer. Ann Oncol.

[3] Mehta RG, Murillo G, Naithani R, Peng X (2010). Cancer chemoprevention by natural products: how far have we come?. Pharm Res.

[4] Neergheen VS, Bahorun T, Taylor EW, Jen LS, Aruoma OI (2010). Targeting specific cell signaling transduction pathways by dietary and medicinal phytochemicals in cancer chemoprevention. Toxicology.

[5] Chen G, Lu F, Xu L, Dong H, Yi P, Wang F, Huang Z, Zou X (2013). The anti-diabetic effects and pharmacokinetic profiles of berberine in mice treated with Jiao-Tai-Wan and its compatibility. Phytomedicine.

[6] Wang J, Qi Q, Feng Z, Zhang X, Huang B, Chen A, Prestegarden L, Li X, Wang J (2016). Berberine induces autophagy in glioblastoma by targeting the AMPK/mTOR/ULK1-pathway. Oncotarget.

[7] Gruenwald J, Freder J, Armbruester N (2010). Cinnamon and health. Crit Rev Food Sci Nutr.

[8] Li H, Li G, Liu L, Guo Z, Ma X, Cao N, Lin H, Han G, Duan Y, Du G (2015). Tumor interstitial fluid promotes malignant phenotypes of lung cancer independently of angiogenesis. Cancer Prev Res.

[9] Pelicano H, Martin DS, Xu RH, Huang P (2006). Glycolysis inhibition for anticancer treatment. Oncogene.

[10] Shackelford DB, Shaw RJ (2009). The LKB1-AMPK pathway: metabolism and growth control in tumour suppression. Nat Rev Cancer.

[11] Turner N, Li JY, Gosby A, To SW, Cheng Z, Miyoshi H, Taketo MM, Cooney GJ, Kraegen EW, James DE, Hu LH, Li J, Ye JM (2008). Berberine and its more biologically available derivative, dihydroberberine, inhibit mitochondrial respiratory complex I: a mechanism for the action of berberine to activate AMP-activated protein kinase and improve insulin action. Diabetes.

[12] Huang B, Yuan HD, Kim DY, Quan HY, Chung SH (2011). Cinnamaldehyde prevents adipocyte differentiation and adipogenesis via regulation of peroxisome proliferator-activated receptor-γ (PPARγ) and AMP-activated protein kinase (AMPK) pathways. J Agric Food Chem.

[13] Izquierdo-Vega JA, Morales-González JA, Sánchez Gutiérrez M, Betanzos-Cabrera G, Sosa-Delgado SM, Sumaya-Martínez MT, Á Morales-González, Paniagua-Pérez R, Madrigal-Bujaidar E, Madrigal-Santillán E (2017). Evidence of some natural products with antigenotoxic effects. Part1: Fruits and Polysaccharides. Nutrients.

[14] Zhou J, Qu Z, Yan S, Sun F, Whitsett JA, Shapiro SD, Xiao G (2015). Differential roles of STAT3 in the initiation and growth of lung cancer. Oncogene.

The article "Berberine and cinnamaldehyde together prevent lung carcinogenesis" was retracted in 2024. Reason: duplicated images.

[15] Cao N, Ma X, Guo Z, Zheng Y, Geng S, Meng M, Du Z, Lin H, Duan Y, Du G (2016). Oral kanglaite injection (KLTI) attenuates the lung cancer-promoting effect of high-fat diet (HFD)-induced obesity. Oncotarget.

[16] Shih JY, Yang PC (2011). The EMT regulator slug and lung carcinogenesis. Carcinogenesis.

[17] Meyskens FL, Mukhtar H, Rock CL, Cuzick J, Kensler TW, Yang CS, Ramsey SD, Lippman SM, Alberts DS (2016). Cancer prevention: obstacles, challenges, and the road ahead. J Natl Cancer Inst.

[18] Che CT, Wang ZJ, Chow MS, Lam CW (2013). Herb-herb combination for therapeutic enhancement and advancement: theory,practice and future perspectives. Molecules.

[19] Qi F, Zhao L, Zhou A, Zhang B, Li A, Wang Z, Han J (2015). The advantages of using traditional Chinese medicine as an adjunctive therapy in the whole course of cancer treatment instead of only terminal stage of cancer. Biosci Trends.

[20] Maresso KC, Tsai KY, Brown PH, Szabo E, Lippman S, Hawk ET (2015). Molecular cancer prevention: current status and future directions. CA Cancer J Clin.

[21] DuBois RN (2006). Cancer prevention: strategy for the future. Carcinogenesis.

[22] Momcilovic M, Bailey ST, Lee JT, Fishbein MC, Magyar C, Braas D, Graeber T, Jackson NJ, Czernin J, Emberley E, Gross M, Janes J, Mackinnon A (2017). Targeted inhibition of EGFR and glutaminase induces metabolic crisis in EGFR mutant lung Cancer. Cell Rep.

[23] Selwan EM, Finicle BT, Kim SM, Edinger AL (2016). Attacking the supply wagons to starve cancer cells to death. FEBS Lett.

[24] Kim SM, Roy SG, Chen B, Nguyen TM, McMonigle RJ, McCracken AN, Zhang Y, Kofuji S, Hou J, Selwan E, Finicle BT, Nguyen TT, Ravi A (2016). Targeting cancer metabolism by simultaneously disrupting parallel nutrient access pathways. J Clin Invest.

[25] Hu K, Gong X, Ai Q, Lin L, Dai J, Cai L, Jiang R, Ge P, Zhang L (2017). Endogenous AMPK acts as a detrimental factor in fulminant hepatitis via potentiating JNK-dependent hepatocyte apoptosis. Cell Death Dis.

[26] Dasgupta B, Milbrandt J (2009). AMP-activated protein kinase phosphorylates retinoblastoma protein to control mammalian brain development. Dev Cell.

[27] Jeon SM (2016). Regulation and function of AMPK in physiology and diseases. Exp Mol Med.

[28] Gailite I, Aerne BL, Tapon N (2015). Differential control of Yorkie activity by LKB1/AMPK and the Hippo/Warts cascade in the central nervous system. Proc Natl Acad Sci USA.

[29] Gomes D, Agasse A, Thiébaud P, Delrot S, Gerós H, Chaumont F (2009). Aquaporins are multifunctional water and solute transporters highly divergent in living organisms. Biochim Biophys Acta.

The article "Berberine and cinnamaldehyde together prevent lung carcinogenesis" was retracted in 2024. Reason: duplicated images.

[30] Zhang Y, Tian K, Wang Y, Zhang R, Shang J, Jiang W, Wang A (2016). The effects of aquaporin-1 in pulmonary edema induced by fat embolism syndrome. Int J Mol Sci.

[31] Tomita Y, Dorward H, Yool AJ, Smith E, Townsend AR, Price TJ, Hardingham JE (2017). Role of aquaporin 1 signalling in cancer development and progression. Int J Mol Sci.

[32] Yokoyama Y, Iguchi K, Usui S, Hirano K (2011). AMP-activated protein kinase modulates the gene expression of aquaporin 9 via forkhead box a2. Arch Biochem Biophys.

[33] Shackelford DB, Shaw RJ (2009). The LKB1-AMPK pathway: metabolism and growth control in tumour suppression. Nat Rev Cancer.

[34] Liang J, Mills GB (2013). AMPK: a contextual oncogene or tumor suppressor?. Cancer Res.

[35] Dahmani R, Just PA, Delay A, Canal F, Finzi L, Prip-Buus C, Lambert M, Sujobert P, Buchet-Poyau K, Miller E, Cavard C, Marmier S, Terris B (2015). A novel LKB1 isoform enhances AMPK metabolic activity and displays oncogenic properties. Oncogene.

[36] Chen G, Lu F, Xu L, Dong H, Yi P, Wang F, Huang Z, Zou X (2013). The anti-diabetic effects and pharmacokinetic profiles of berberine in mice treated with Jiao-Tai-Wan and its compatibility. Phytomedicine.

[37] Zou X, Huang W, Lu F, Fang K, Wang D, Zhao S, Jia J, Xu L, Wang K, Wang N, Dong H (2017). The effects of Jiao-Tai-Wan on sleep, inflammation and insulin resistance in obesity-resistant rats with chronic partial sleep deprivation. BMC Complement Altern Med.

[38] Huang Z, Xu X, Lu F, Wang N, Chen G, Zhao Y, Zou X, Wang K, Dong H, Xu L (2013). Jiao tai wan attenuates hepatic lipid accumulation in type 2 diabetes mellitus. Evid Based Complement Alternat Med.

[39] Hamet P (1996). Cancer and hypertension. An unresolved issue. Hypertension.

[40] Giovannucci E, Harlan DM, Archer MC, Bergenstal RM, Gapstur SM, Habel LA, Pollak M, Regensteiner JG, Yee D (2010). Diabetes and cancer: a consensus report. Diabetes Care.

[41] Ma X, Deng J, Cao N, Guo Z, Zheng Y, Geng S, Meng M, Lin H, Duan Y, Du G (2016). Lasting glycolytic stress governs susceptibility to urethane-induced lung carcinogenesis in vivo and in vitro. Toxicol Lett.

[42] Zhou JY, Zhou SW, Zhang KB, Tang JL, Guang LX, Ying Y, Xu Y, Zhang L, Li DD (2008). Chronic effects of berberine on blood, liver glucolipid metabolism and liver PPARs expression in diabetic hyperlipidemic rats. Biol Pharm Bull.

[43] Ma YG, Zhang YB, Bai YG, Dai ZJ, Liang L, Liu M, Xie MJ, Guan HT (2016). Berberine alleviates the cerebrovascular contractility in streptozotocin-induced diabetic rats through modulation of intracellular Ca2+ handing in smooth muscle cells. Cardiovasc Diabetol.

[44] Singh A, Khan SA, Choudhary R, Bodakhe SH (2016). Cinnamaldehyde attenuates cataractogenesis via restoration of hypertension and oxidative stress in fructose-fed hypertensive rats. J Pharmacopuncture.

The article "Berberine and cinnamaldehyde together prevent lung carcinogenesis" was retracted in 2024. Reason: duplicated images.

[45] Taguchi Y, Hayama K, Okada M, Sagawa T, Arai R, Abe S (2011). Therapeutic effects of cinnamaldehyde and potentiation of its efficacy in combination with methylcellulose on murine oral candidiasis. Med Mycol J.

[46] Liu L, Li H, Guo Z, Ma X, Cao N, Zheng Y, Geng S, Duan Y, Han G, Du G (2015). The combination of three natural compounds effectively prevented lung carcinogenesis by optimal wound healing. PLoS One.

